The article "3D Automatic Segmentation of Brain Tumor Based on Deep Neural Network and Multimodal MRI Images" was retracted in 2023. Reasons: signs of a paper mill; suspected computer-generated content; unreliable results or conclusions; lack of ethics approval or compliance.

# 3D Automatic Segmentation of Brain Tumor Based on Deep Neural Network and Multimodal MRI Images

**DOI:** 10.1155/2022/5356069

**Published:** 2022-08-21

**Authors:** Zhuliang Qian, Lifeng Xie, Yisheng Xu

**Affiliations:** Department of Imaging, Xiaoshan District Hospital of Traditional Chinese Medicine, Hangzhou 311201, Zhejiang, China

## Abstract

Brain tumor segmentation is an important content in medical image processing, and it is also a very common research in medicine. Due to the development of modern technology, it is very valuable to use deep learning (DL) and multimodal MRI images to study brain tumor segmentation. In order to solve the problems of low efficiency and low accuracy of brain tumor segmentation, this paper proposes DL to conduct research on multimodal MRI image segmentation, aiming to make accurate diagnosis and treatment for doctors. In addition, this paper constructs an automatic diagnosis system for brain tumors, uses GLCM and discrete wavelet transform (DWT) to extract features from MRI images, and then uses a convolutional neural network (CNN) for final diagnosis; finally, through four. The comparison of the results between the two algorithms proves that the CNN algorithm has the better processing power and higher efficiency.

## 1. Introduction

In recent years, through quantitative analysis of a large number of medical images, the relationship between the features contained in these images and their respective diseases has been discovered, and some progress has been made in automated omics imaging methods. Automatic classification is of great significance to the diagnosis of diseases. With the successful application of imaging in clinical medicine, quantitative analysis of imaging will play an increasingly important role in imaging. When classifying the volume image, in order to facilitate subsequent processing and segmentation results, the tumor part needs to be separated from the image to affect the subsequent processing of the information. The reliance on manual fragmentation is time-consuming and painful, mainly depends on the operator, and may lead to the loss of some useful information. Therefore, it is very important to study the automatic segmentation method of tumor images.

When the receiver is equipped with a limited number of radio frequency (RF) chains in a beam space millimeter wave (mmWave) large-scale multiple-input and multiple-output system, the channel estimation will be very challenging. To solve this problem, He H uses a learning-based noise reduction-based approximate message passing (LDAMP) network. The neural network can learn the channel structure and estimate the channel from a large amount of training data. However, the efficiency of DL in the communication process is not very high [1]. Brain tumor segmentation is the process of separating the tumor from the normal brain tissue. Michael's research introduced a new segmentation algorithm called DeepJoint segmentation and multiclassifier to classify the severity of glioma tumors. Initially, the brain image is preprocessed, and then the region of interest is extracted. Then, use the suggested DeepJoint segmentation to complete the segmentation of the preprocessed image. After segmentation, information theory methods are used to extract features from core and edema tumors. Finally, classification is performed by a deep convolutional neural network (DCNN), which is trained by an optimization algorithm called Fractional Jaya Whale Optimizer (FJWO). However, there are some errors in the segmentation process of multimodal MRI images, resulting in inaccurate results [2]. Sérgio Pereira proposed an automatic segmentation method based on CNN and explored 3 × 3 small cores. Considering that there are fewer weights in the network, using a small kernel can design a deeper architecture, in addition to having a positive effect on overfitting. However, the complexity of the segmentation method is too high, leading to errors in the results [3].

The innovations of this article are (1) Magnetic resonance imaging (MRI) is a commonly used auxiliary diagnostic tool for brain diseases. It has the advantages of noninvasive, harmless to the human body, and high soft tissue resolution. Magnetic resonance imaging, as a multiparameter imaging method, has a high sensitivity to the display of tissue morphology and pathological changes. (2) Brain tumor segmentation plays an important role in assisting doctors in diagnosis and formulating treatment plans. The goal is to segment abnormal brain tissues.

## 2. Brain Tumor Segmentation Method Based on DL and Multimodal MRI Images

### 2.1. Automatic Diagnosis Method of Brain Tumor

#### 2.1.1. DWT

After performing a two-dimensional discrete wave transformation on each image, an approximate low-pass sub-region and three high-pass sub-regions representing detailed information can be used. The four sub-regions are marked as LL, LH, HH, and HL. HH, HL, and LH, respectively, correspond to the high-frequency part of the image and reflect the detailed information of the image. LL corresponds to the low-frequency part of the image. The two parts, respectively, contain most of the energy information in the image [4, 5]. The two-dimensional discrete wave transform can repeat the discrete wave transform in the low-frequency sub-region, which can obtain any decomposition from the formula to obtain the decomposition of multiple analyses. In the experiment, considering the accuracy of calculation and classification, we only perform a one-level decomposition of the initial image. Since the main image information is concentrated in the low-frequency range (by comparison, it can be seen that the low-frequency sub-region has a good visual effect and is almost too close to the original image), the gray coexistence table is calculated in the low-frequency subset. Since the high-frequency part also contains some image features, it cannot be rejected immediately. Therefore, the change of the transformation factor is calculated in the high-frequency and low-frequency sub-regions of the image as a statistical feature [6, 7].

#### 2.1.2. GLCM

GLCM is obtained by counting the number of occurrences of pixel pairs in a certain direction and a distance of *d* in the image. The GLCM takes into account the number of pixels in the image, factors such as the grayscale relationship, spatial distance, and mutual direction [8, 9]. Furthermore, the texture information can be represented by a relative frequency matrix. This frequency is the number of times two pixels with a distance of *d* appear on the entire image. The GLCM can be expressed as a function of two pixels with a distance of *d* in a certain direction and the positional relationship between the gray values of related pixels [10, 11]. In order to reflect the probability of pixel pairs appearing on the entire image, according to the literature, this frequency relative matrix needs to be normalized, and the normalization process is carried out according to formulas (1) and (2) [12, 13]. Normalization is a dimensionless processing method that turns the absolute value of the physical system value into a relative value relationship.

(1) $$\begin{array}{c} p\left(i,j\right)=\frac{T\left(i,j\right)}{R}. \end{array}$$

(2) $$\begin{array}{c} R=\left\{\begin{array}{c} 2a\left(b-d\right),\theta =0^{\circ }\text{ or }\theta =90^{\circ },\\ 2\left(b-d\right)\left(a-d\right),\theta =45^{\circ }\text{ or }\theta =135^{\circ }. \end{array}\right) \end{array}$$

Among them, *D* is the distance between two pixels with gray value *i* and gray value *j*, a is the number of rows in the original image, *b* is the number of columns in the original image, and *R* represents the occurrence of all pairs of pixels with a spacing of *d* in the *θ* direction The total number of times, *θ* is the four directions when calculating GLCM.

Figure 1 shows the specific implementation process of the feature extraction method in this chapter [14]. After the image undergoes two-dimensional DWT, the GLCM and variance are calculated in the low-frequency part; in order to obtain the rotation invariant characteristics of the high-frequency part, the three high-frequency parts are added together to find the variance in the experiment [15, 16]. Finally, the three are connected together as the texture feature of the image.

#### 2.1.3. CNN

CNN is a special model of a deep neural network. The structure of this network is inspired by the neural mechanism of the optical system. It is a multilayer perceptron specially designed to recognize two-dimensional shapes [17]. The convolutional neural network is constructed by imitating the visual perception mechanism of biology and can grid features with a small amount of calculation. The main neural network generally consists of an input layer, an aggregation layer, a down-sampling layer (concentration layer), a fully connected mattress, and an outlet mattress.

The basic structure of CNN consists of two parts: among them, the feature extraction layer is used to extract local regional features, and the input of each neuron is related to its local receptor field. After deriving a local attribute, it is necessary to determine its relationship with other local attributes. The second is the feature mapping level. Each layer of the computer in the network consists of many feature maps, and each feature map is flat, and the weights of all neurons at this level are equal [18, 19]. The feature map structure uses the Sigmoid function with a small influence function kernel as the activation function of the convolution network, so that the feature map has displacement invariance.

The convolutional layer is the main component of CNN. The definition of subsequent operations is as follows:

(3) $$\begin{array}{c} C_{ij}=\sum_{s=1}^{p}\sum_{t=1}^{q}a_{i+p-s,j+q-t}•b. \end{array}$$

Among them, the size of matrix A is P ^*∗*^ Q, and the size of matrix B is expressed by p ^*∗*^ q. Each element in their convolution C can be calculated by the above formula.

#### 2.1.4. Classification of Sparrow Search Algorithms (ESSAs)

In the standard sparrow search algorithm, when the values of the inertia factor *w*_*n*_ for inducing motion and the inertia factor*w*_*h*_ for foraging motion are large, it is helpful for the algorithm to avoid falling into the local minimum, thereby improving the global search ability; when the two factors have relatively high values it is helpful to improve the algorithm's ability to search for the local area where the sparrow is currently located; therefore, it can be known that a reasonable adjustment of the value of a factor is the key to improving the performance of the algorithm. In order to improve the convergence speed and accuracy of the algorithm, this paper proposes a sparrow search algorithm that dynamically adjusts the inertia weight. The inertial weight decreases linearly with the increase in the number of repetitions. It effectively prevents the decline of local search capabilities and has significant advantages in local and global search capabilities. The improvement strategy is

(4) $$\begin{array}{c} w_{n}=w_{h}=\frac{xsd\left(i,j\right)+w_{\min}-w_{\max}}{t_{\max}}\left(t_{\max}-t\right), \end{array}$$

Among them, *xsd*(*i*, *j*) ∈ (0,1) represents the similarity value of krill individuals *i* and *j* in the krill population, *t* represents the current iteration number, *t*_max_ represents the maximum iteration number, and *w*_max_ represents the induced inertia factor and foraging. The maximum value of the inertia factor and *w*_min_ represents its minimum value [20]. This improvement strategy allows the two factors of the algorithm to be adjusted according to the current krill population situation, which can effectively adjust the algorithm's global search and local survey capabilities. However, in practical applications, this linear reduction of information strategy exists locally in the initial stage of replication. The shortcomings of weak research ability and weak global ability; search in the later stage of the repetition. This will make the best points in the world easy to lose at the beginning of the repetition, and local optimization in the later price stage [21]. Aiming at the shortcomings of the linear decreasing update strategy, this paper continues to study the influence of the inertia weight on the algorithm based on it, in order to further improve its convergence speed and accuracy, and proposes an improved sparrow search optimization algorithm (IKHA). Here is a time-varying nonlinear decrement strategy, namely:

(5) $$\begin{array}{c} w_{n}=w_{h}=w_{\min}*\text{rand}+\left(w_{\text{max}}-w_{\text{min}}\right)\left(2-e^{\text{log}\left(2\right)*t/MI}\right). \end{array}$$

In the formula, MI represents the current maximum number of iterations [22, 23]. This strategy makes the overall algorithm *w*_max_ and*w*_min_ gradually decrease, allowing the algorithm to better adjust the current search capability during the entire optimization process to avoid falling into the local optimal value, thereby further improving the algorithm's global search capability and convergence speed (the speed at which a convergent sequence approaches its limit).

The optimization process of the Improved Sparrow Search Optimization Algorithm (IKHA) can be described as follows:

(6) $$\begin{array}{c} X_{i}\left(t+\Delta t\right)=X_{i}\left(t\right)+\Delta t\frac{dX_{i}}{dt}+r1\left(X_{\text{best}}\left(t\right)-X_{i}\left(t\right)\right). \end{array}$$

### 2.2. Principles of MRI Imaging

Magnetic imaging is based on the quantum mechanical properties of proton rotation, such as electrons and atomic nuclei, which also have angular momentum. The specific value of the angular torque should be determined according to the quantum torque of the magnetic core. Magnetic resonance imaging is an imaging technology that uses the signal generated by the resonance of atomic nuclei in a strong magnetic field to reconstruct the image. It is a nuclear physical phenomenon. In different magnetic fields, such as the brain, protons can be excited to generate radio frequency signals, and this signal can be recognized by the receiving circuit [24]. At present, only atomic nuclei whose rotation quantum number is equal to 1/2 can identify the NMR signal of the receiving circuit.

The most commonly used MRI scan is from a spin echo imaging sequence. The image input in this order is a function of two parameters of the instrument, one parameter is coordination time (TD), and the other is repetition time (TR). MRI can obtain images of the body's transverse, coronal, sagittal, and cross-sections in any direction, which is beneficial to the three-dimensional localization of lesions. An image blood vessel in the MR-wing image represents the nuclear magnetic coordination signal of the volume element hydrogen in the body. The image of the MR image of the body tissue can be expressed by the following equation:

(7) $$\begin{array}{c} S\left(TR,TE\right)=\sum {}_{i}p_{i}\left(1-e^{-\left(TR/t1_{i}\right)}\right)\left(e^{-TE/t2_{i}}\right). \end{array}$$

Among them, *t*1 is the rotation relaxation time, also known as the relaxation length time, which reflects the time required for the switch core to transfer the absorbed energy to the surrounding power grid. It is also the time required for the 90 RF pulsed proton to recover to its original state before the magnetism is triggered. *t*2 is the torque rotation relaxation time, also known as the transverse relaxation time, which reflects the decomposition and loss process of transverse magnetism [25]. The weakening of *T*2 is caused by the mutual magnetization between coordinating protons, which is different from *t*1 which causes the phase change. *p* is the density of the rotation type in the voxel.

The proton is positively charged and continues to rotate around its axis like the Earth, generating its own magnetic field. Generally speaking, the arrangement of the rotation axis of the small magnet is unstable and chaotic, but if a strong external magnetic field is applied, the rotation axis of the small magnet should be rearranged according to the direction of the magnetic force line. When protons are in a chaotic state, and now they are placed in a strong external magnetic field, the split state of the protons will change. It only points in two directions parallel or antiparallel to the external magnetic field. If it is stimulated by a pulse of a specific frequency, it will be used as a small magnet. The hydrogen core of the magnet absorbs a certain amount of energy and resonance, that is, magnetic coordination occurs.

### 2.3. Brain Tumor Segmentation Method

#### 2.3.1. FCM Segmentation Method

Fuzzy clustering method (FCM) is an unsupervised classification method, which is widely used in brain tumor image segmentation. The FCM clustering method is based on the minimization of the objective function (the form of the goal pursued in terms of design variables), which becomes the c-mean function.

(8) $$\begin{array}{c} J\left(X;U,V\right)=\sum_{i=1}^{c}\sum_{a=1}^{N}{\left(u_{ia}\right)}^{m}{\left\|x_{a}-v_{i}\right\|}_{A}^{2}. \end{array}$$

(9) $$\begin{array}{c} D_{\text{iaA}}^{2}={\left\|x_{a}-v_{i}\right\|}_{A}^{2}={\left(x_{a}-v_{i}\right)}^{t}A\left(x_{a}-v_{i}\right). \end{array}$$

For the data *X*=[*x*_1_, *x*_2_,…, *x*_*n*_],  *x*_*i*_ ∈ *R*^*s*^, *s* is the number of features and *V*=[*v*_1_, *v*_2_,…, *v*_*n*_] is the prototype of geometric clustering. *u*_*ia*_ stands for cluster center, and*v*_*i*_ is *c* prototype. The number of classes *c* must be given, and*D*_iaA_^2^ is the cluster center of each region. The stagnation point of the objective function can also be found by the following formula:

(10) $$\begin{array}{c} \overset{-}{J}\left(X;U,V,\rho \right)=\sum_{i=1}^{c}\sum_{a=1}^{N}{\left(u_{ia}\right)}^{m}D_{\text{iaA}}^{2}+\sum_{a=1}^{N}\rho_{a}\left(\sum_{i=1}^{c}u_{ia}-1\right). \end{array}$$

The minimization of $\overset{-}{J}$ is based on the appropriate selection of *U* and *V* through the following formula:

(11) $$\begin{array}{c} u_{ia}=\frac{1}{\sum_{j=1}^{c}{\left(D_{\text{iaA}}/D_{\text{jaA}}\right)}^{2/\left(m-1\right)}},\;1\leq i\leq c,\;1\leq a\leq n. \end{array}$$

(12) $$\begin{array}{c} v_{i}=\frac{\sum_{a=1}^{n}u_{ia}^{m}x_{a}}{\sum_{a=1}^{n}u_{ia}^{m}},1\leq i\leq c. \end{array}$$

The algorithm can be summarized in the following steps:

(1) Give the number of clusters *c*, the weight index *m*, the norm induction matrix *A*, and the termination tolerance *e*.
(2) Initialize the segmentation matrix *U*.
(3) Use *U* and the formula *v*_*i*_ to calculate the cluster prototype.
  (13) $$\begin{array}{c} v_{i}^{\left(l\right)}=\frac{\sum_{a=1}^{N}u_{ia}^{\left(l-1\right)}x_{a}}{\sum_{a=1}^{N}{\left(u_{ia}^{\left(l-1\right)}\right)}^{m}},1\leq i\leq c. \end{array}$$
(4) Calculate the distance as
  (14) $$\begin{array}{c} D_{\text{iaA}}^{2}={\left(x_{a}-v_{i}\right)}^{t}A\left(x_{a}-v_{i}\right),\;1\leq i\leq c;1\leq a\leq N. \end{array}$$
(5) Update distance as

(15) $$\begin{array}{c} v_{i,a}^{\left(l\right)}=\frac{1}{\sum_{j=1}^{c}{\left(D_{\text{iaA}}/D_{\text{jaA}}\right)}^{2/\left(m-1\right)}}, \end{array}$$

until

(16) $$\begin{array}{c} \left\|U^{\left(l\right)}-U^{\left(l-1\right)}\right\|<e. \end{array}$$

#### 2.3.2. Gaussian Kernel Fuzzy C-Means Clustering

The commonly used Gaussian Kernel Fuzzy C-Means Clustering Algorithm (KFCM) can be divided into KFCM-1 algorithm and KFCM-2 algorithm. Here, we mainly introduce the KFCM-1 algorithm. This method forms a mapping relationship through the kernel function, converts the points in the original space to the feature space for calculation and analysis, and finally obtains the optimal division of the original space. The main idea of the KFCM-1 algorithm is to use the kernel function to transform the data from a low-dimensional feature space into a high-dimensional feature space, so that the features that were not well displayed can be displayed and the difference between different categories is improved. This method is somewhat similar to the solution of a support vector machine (SVM). Support vector machines use kernel tricks to classify nonlinear data. When supervised learning is not possible and the numbers are not labeled, data clustering is used to classify the data. At this time, the learning is unsupervised and the support vector clustering algorithm is used. The specific mathematical description is that there are generally two steps for clustering in the feature space. First, transform the space to a high-dimensional space F through a nonlinear mapping *ο* : *λ*⟶*F*(*x* ∈ *R*^*p*^⟶*ο*(*λ*)),  *q* > *p*, and then cluster in the space *F*. Comparing the expression form of the low-dimensional cluster center, we can remember the cluster center in the high-dimensional space *F* as *d*_*i*_ as follows:

(17) $$\begin{array}{c} d_{i}=\sum_{j=1}^{n}\beta_{ij}ο\left(x_{j}\right),\;\forall i=1,2,\ldots ,n. \end{array}$$

The objective function of KFCM-1 is as follows:

(18) $$\begin{array}{c} J_{m}\left(U,d\right)=J_{m}\left(U,\beta_{1},\beta_{2},\ldots ,\beta_{d}\right)=ο{\left(x_{j}\right)}^{T}ο\left(x_{j}\right)-23\sum_{l=1}^{n}\beta_{il}{\left(x_{l}\right)}^{T}ο\left(x_{j}\right)+\sum_{l=1}^{n}\sum_{k=1}^{n}\beta_{il}{\left(x_{j}\right)}^{T}ο\left(x_{j}\right). \end{array}$$

The calculations in (18) are all in the form of the inner product of the elements. The inner product is a vector operation, that is, the corresponding elements are multiplied and added, and the result is a scalar.

## 3. Construction Experiment of Brain Tumor Automatic Diagnosis Auxiliary System Based on Multimodal MRI Images

### 3.1. Computer-Aided System for Automatic Diagnosis of Brain Tumors

The workflow of the computer-aided system for the automatic diagnosis of brain tumors is shown in Figure 2. A preprocessing device-automatic smear device is used in the system to make cell smears used in the test, which is an auxiliary device of this system. The system adopts modular design ideas, each module is closely related to other modules, and connects up and down.

In traditional micro preparation, the doctor artificially melts the cell sample into a glass plate. Recent studies have shown that the coating made by this traditional manual method can only collect 20% of the cells, while more than 80% of the cell samples remain in the sample and are discarded together. In addition, more than 40% of the coating will become turbid due to the action of blood, mucus, and inflammatory tissue. These defects are the reason for the inaccurate results of most routine tests. The automation of cell smears not only improves the efficiency of the system, but also ensures the consistency of the system and the standardization of cell staining, thereby reducing the difficulty of identifying machines and improving the correct identification rate. The task of the pretreatment equipment is to automatically prepare cell staining. The working procedure of the instrument is as follows: using the principle of adsorption, diluting the cell sampling with a diluent, then uniformly stirring and filtering with an appropriate semipermeable membrane, staining with an appropriate staining method, forming a very thin cell coating on the window pane, use a fixative for fixation, and finally a drying process, coating extremely thin cells, the cell shape is well preserved and evenly distributed.

The computer-aided diagnosis instrument shall include microscopic visual inspection devices and automatic identification software. One is the foundation of the inspection system, and the other is the core and key of the inspection system. The two complement each other and are indispensable. The material system mainly includes an optical microscope, a precision workbench, an optical collection device, and a computer. The software system mainly includes image algorithm modules, cell segmentation (including core and coil segmentation) modules, export characteristics, and analysis and identification. Under the coordinated control of the computer, the unit controller drives the desktop to scan in the *X* and Y directions and focus correction in the *Z* direction. The CCD camera collects clear images of the cells magnified by the microscope and transmits them to the computer for processing and analysis.

### 3.2. Brain Tumor Segmentation Processing Steps

Magnetic resonance image preprocessing is a very active research area, which is dedicated to improving and correcting magnetic resonance images for future analysis. In the unsupervised method, the brain tissue data learning model without reference or nonauto-labeling will encounter common problems such as noise or gray inconsistency, which will cause the system to accumulate errors as the error categories increase. MRI brain tumor segmentation usually follows the following steps:

Denoising is a typical work of magnetic imaging preprocessing, its purpose is to reduce or ideally eliminate noise in the original magnetic imaging image. Although MRI noise is usually Gaussian, by definition, MRI noise generally obeys the Rician distribution. The main source of MRI image noise is the detection object, mainly thermal noise, and sometimes physiological noise.

Skull dissection is the process of removing the skull, hemorrhage, and nonbrain tissue from the MRI sequence. Brain Suite software can be used to improve data preprocessing, recalculate the autopsy masks of all patients, and delete unnecessary tissues in MRI images.

Abnormal intensity is another common artificial target during MRI data acquisition. Magnetic field anomalies are an inevitable result, including low-frequency signals destroying images and affecting grayscale. Grayscale uses black tones to represent objects, that is, black is used as the base color, and black with different saturations is used to display images.

In brain tumor injury plans, many magnetic imaging sequences are usually obtained through different analyses. Furthermore, introducing spatial inconsistency in multiple MRI studies.

### 3.3. Feature Extraction

There is a high degree of correlation between adjacent voxels in medical images, and the grayscale patterns between adjacent voxels are different, and the volumes are the same. This method uses patch prediction based on small image regions, which can make full use of these local correlation information, and can predict a set of limited image block vocabularies based on small image regions. This method has been widely used in the fields of image denoising, image reconstruction, and image pattern synthesis. This method converts the image segmentation problem into the image unit classification problem by predicting the most likely label category of the central image unit and has achieved great success. All methods are similar to this focus on the study of the similarity between unnecessary local image information and its image features in near pixels. This article directly derives the target image and the small-area *m* and organizes them as features in the form of a one-dimensional vector *m* × m × *m*.

Due to the imbalance between volume samples and nonvolume samples, a sampling method is used to reduce the positive and negative samples to 10 W data volume for training.

### 3.4. Results Evaluation

This experiment uses the training and testing data set provided by BRATS2015. In order to evaluate the performance of algorithm segmentation, the segmentation results are uploaded to the online evaluation system of the competition. Four indicators of Dice score, PPV, Sensitivity, and Kappa are used to evaluate the performance. The relevant definitions are as follows:

(19) $$\begin{array}{c} \text{Dice}\left(U,V\right)=\frac{2\left(\left|U_{1}\cap V_{1}\right|\right)}{\left|U_{1}\right|+\left|V_{1}\right|}. \end{array}$$

(20) $$\begin{array}{c} \text{ppv}\left(U,V\right)=\frac{\left(U_{1}\cap V_{1}\right)}{\left|V_{1}\right|}. \end{array}$$

(21) $$\begin{array}{c} \text{sensi}\left(U,V\right)=\frac{\left(U_{1}\cap V_{1}\right)}{\left|U_{1}\right|}. \end{array}$$

(22) $$\begin{array}{c} \text{Kappa}\left(U,V\right)=\frac{\left|U⊕V\right|/\left|U_{0}+V_{1}\right|-\left|U_{0}\right|•\left|V_{0}+\left|U_{1}\right|•\left|V_{1}\right|\right|/\left(\left|U_{0}\right|+\left|V_{0}\right|\right)•\left(\left|U_{1}\right|+\left|V_{1}\right|\right)}{\left|U_{0}\right|•\left|V_{0}\right|+\left|U_{1}\right|•\left|V_{1}\right|/\left(\left|U_{0}\right|+\left|V_{0}\right|\right)•\left(\left|U_{1}\right|+\left|V_{1}\right|\right)}. \end{array}$$

*G* represents the result of manual segmentation by experts, and *S* represents the result of segmentation by the algorithm in this chapter. U0 and U1 are manually divided into negative and positive samples. Similarly, *V*0 and *V*1, respectively, represent the negative and positive samples predicted by the algorithm.

## 4. Brain Tumor Segmentation Algorithm Based on Machine Learning and Multimodal MRI Images

### 4.1. Brain Tumor Segmentation Algorithm Based on Multimodal MRI Images

This article uses some segmented MR images in the public data set in the Whole Brain Atlas (WBA) database as training data. The first part shows the segmentation results on the No. 4 instance of the high-level whole brain Atlas WBA_TA; the second part is the segmentation results on the No. 20 instance of the low-level whole brain Atlas WBA_TB. Divide between*W*1 and *W*2, W1C, and WBA numbers.

This paper evaluates the segmentation efficiency of the algorithm based on the measurement of the Dice factor. The measured value of the Dice factor is in the range of [0,1], where 1 means a perfect match, and 0 means a complete disagreement. Use the training data set to simulate 20 WBA-TA and 20 WBA-TB instances, and record the measured value of the Dice factor.  Table 1 and Figure 3, respectively, correspond to the results of 8 simulation examples.

Comparing the algorithm in this article with the current three technologies, Table 2 and Figure 4 list the average results of measuring the dice factors of these algorithms used to split the image into the data set. It can be seen that the algorithm in this paper achieves the best results when segmenting the volume and the volume of different images.

In addition, many existing segmentation algorithms require additional model training, so it takes a lot of time and depends on a specific training set. This algorithm realizes volume segmentation based on gray distribution matching and does not require manual calibration of large amounts of data for model training, which effectively reduces segmentation time. Experiments show that the average segmentation time of this algorithm for each image is about 0.5 s. For some automatic segmentation algorithms that do not require training, the segmentation time of these algorithms is close to or slightly less than the algorithm in this article, but its segmentation accuracy is also obvious lower. In practical applications, the accuracy of subdivision is more important than the time of division. In short, the algorithm proposed in this paper significantly improves the accuracy of the segmentation while keeping the segmentation time low.

### 4.2. Results and Analysis of Brain Tumor Image Segmentation Based on MRI

This experiment uses a synthetic MRI data set with fewer artifacts and grayscale variables compared with real MRI images. This verification experiment does not include rough extraction.

The experiment uses an image patch with a size of 3 × 3 × 3, and the dictionary atomic sequence *K* = [2 4 8 16 32 64 128 256 512] is used to test and explore the optimal *K* value. As shown in Figure 5, as the number of dictionary atoms increases, the average accuracy of segmentation increases very rapidly, and the accuracy does not stabilize until *K* = 128.

In order to compare the average segmentation performance of the segmentation method proposed in this article on the training data set and the test data set, the four indicators of the two are counted and calculated. Among them, the segmentation method proposed in this article is in the training data set of BRATS 2019; the average segmentation performance of the above is shown in Table 3 and Figure 6.

In addition, the average segmentation performance of the segmentation method proposed in this paper on the BRATS 2019 test data set is shown in Table 4 and Figure 7.

According to the requirements of the BRATS competition, the experiment has three different segmentation tasks: complete tumor area R1 (label 1 + 2+3 + 4), tumor core area R2 (label 1 + 3+4), enhanced tumor area R3 (label 4). According to the comparison of the results of the algorithm segmentation in this paper, the segmentation method adopted in this paper has great potential.

## 5. Conclusions

The medical imaging scan of the MRI brain has a high degree of correlation between the target and neighboring voxels, as well as the grayscale calculation of different image modes between the same data volume. The prediction method using small-area image coding can make full use of this locally relevant information can be based on a limited set of image block vocabularies. This paper successfully applies these methods to image segmentation operations by providing the most likely label of the central pixel of the image block. This method focuses to a large extent on exploring the similarity information of the features of adjacent regions of the image.

This article mainly focuses on the uneven grayscale in the segmentation of MRI brain tumor images and the large differences in the size, location, and structure of brain tumors in different patients, such as the large differences in MRI images of different patients. Starting from the segmentation of the entire tumor structure, to the detailed description of the tumor substructure, the self-organizing active contour model and neural decoding network technology are introduced into the segmentation problem based on changeable images, and then the automatic tissue mapping based on the changeable MRI image and the deep deconvolution neural network hybrid active mapping model of brain tumors are proposed Segmentation strategy.

Tumor cell-assisted visual diagnosis system is an important application of computer automatic visual inspection in medical image processing. Based on the analysis of the clinical diagnosis of pathologists, and referring to the results and experience of previous studies, this article conducts an in-depth study on the principle of visual detection of microscopic cell smears, and proposes a set of implementation plans for a tumor cell-assisted diagnosis system. Based on the scheme, a preliminary software identification system is given. Focusing on cell image preprocessing, segmentation, cell classification, and identification, etc., this article has done a lot of research and achieved good preliminary research results. There is still room for improvement in the method in this paper. This paper deals with two-dimensional data. Subsequent work will extend the method to three-dimensional and further optimize the segmentation results.

## Figures and Tables

**Figure 1:** Feature extraction process based on GLCM.

**Figure 2:** Work flow chart of the brain tumor automatic diagnosis system.

**Figure 3:** Dice coefficient metrics for image segmentation.

**Figure 4:** The mean value of the dice coefficient measurement of each segmentation algorithm.

**Figure 5:** The number of dictionary atoms and the accuracy of segmentation.

**Figure 6:** The average correct rate of 200 patients in the training data set with segmentation.

**Figure 7:** The average correct rate with the segmentation of 100 patients in the tested data set.

**Table 1:** Dice coefficient metrics for image segmentation.

Numbering	1	2	3	4	5	6	7	8
WBA_TA-tumor	0.942	0.933	0.904	0.866	0.968	0.854	0.954	0.964

WBA_TA-edema	0.912	0.844	0.925	0.909	0.929	0.555	0.951	0.879

WBA_TB-tumor	0.954	0.800	0.815	0.933	0.905	0.912	0.872	0.821

WBA_TB-edema	0.954	0.850	0.890	0.920	0.900	0.917	0.895	0.644

**Table 2:** The mean value of the dice coefficient measurement of each segmentation algorithm.

Different algorithms	FCM	KFCM	CNN	Algorithm
WBA_TA-tumor	0.72	0.61	0.69	0.88
WBA_TA-edema	0.70	0.64	0.57	0.83
WBA_TB-tumor	0.65	0.48	0.72	0.87
WBA_TB-edema	0.43	0.33	0.39	0.81

**Table 3:** The average correct rate of 200 patients with segmentation in the training data set.

Validation	HGG	LGG
Dice-complete	0.86	0.80
Dice-core	0.76	0.64
Dice-enhancing	0.83	0.73
PPV-complete	0.95	0.83
PPV-core	0.72	0.57
PPV-enhancing	0.81	0.77
Sensitivity-complete	0.75	0.83
Sensitivity-core	0.79	0.76
Sensitivity-enhancing	0.84	0.66
Kappa	1.00	1.00

**Table 4:** The average correct rate with the segmentation of 100 patients in the tested data set.

Split task	Dice	PPV	Sensitivity	Kappa
Complete	0.84	0.83	0.80	1.00
Core	0.71	0.77	0.78	1.00
Enhancing	0.59	0.60	0.66	1.00

## Data Availability

No data were used to support this study.
